The article "Effective Face Detector Based on YOLOv5 and Superresolution Reconstruction" was published in 2021. Journal: Comput Math Methods Med.

# Effective Face Detector Based on YOLOv5 and Superresolution Reconstruction

**DOI:** 10.1155/2021/7748350

**Published:** 2021-11-16

**Authors:** Qingqing Xu, Zhiyu Zhu, Huilin Ge, Zheqing Zhang, Xu Zang

**Affiliations:** School of Electronic Information, Jiangsu University of Science and Technology, Zhenjiang 212003, China

## Abstract

The application of face detection and recognition technology in security monitoring systems has made a huge contribution to public security. Face detection is an essential first step in many face analysis systems. In complex scenes, the accuracy of face detection would be limited because of the missing and false detection of small faces, due to image quality, face scale, light, and other factors. In this paper, a two-level face detection model called SR-YOLOv5 is proposed to address some problems of dense small faces in actual scenarios. The research first optimized the backbone and loss function of YOLOv5, which is aimed at achieving better performance in terms of mean average precision (mAP) and speed. Then, to improve face detection in blurred scenes or low-resolution situations, we integrated image superresolution technology on the detection head. In addition, some representative deep-learning algorithm based on face detection is discussed by grouping them into a few major categories, and the popular face detection benchmarks are enumerated in detail. Finally, the wider face dataset is used to train and test the SR-YOLOv5 model. Compared with multitask convolutional neural network (MTCNN), Contextual Multi-Scale Region-based CNN (CMS-RCNN), Finding Tiny Faces (HR), Single Shot Scale-invariant Face Detector (S3FD), and TinaFace algorithms, it is verified that the proposed model has higher detection precision, which is 0.7%, 0.6%, and 2.9% higher than the top one. SR-YOLOv5 can effectively use face information to accurately detect hard-to-detect face targets in complex scenes.

## 1. Introduction

Face detection is indispensable for many visual tasks and has been widely used in various practical applications, such as intelligent surveillance for smart cities, face unlocking in smartphones, and beauty filters. However, face detection still has many challenges due to the interference of shooting angle, background noise, image quality, face scale, and other factors. In practical scenarios, the missing detection problem of small-scale faces results in poor performance of former face detectors. Thus, many scholars have launched researches on blurring small-size human faces.

Over the past decades, convolutional neural networks (CNNs) have been certified to be useful models for processing a wide range of visual tasks, and we have witnessed the rapid development of general object detectors. The commonly used target detection framework is divided into two branches [1], two-stage detectors and one-stage detectors. Typical algorithms of two-stage detectors include faster R-CNN [2], PANet [3], SPPNet [4], and Mask R-CNN [5]. The second is one-stage detectors, derived from SSD [6], YOLOv1 to YOLOv5 [7–11], and RetinaNet [12]. The former has higher detection accuracy, but its detection speed is slower, while the latter improves the detection speed and maintains performance. At the same time, the design of face detector gain has achieved the state-of-the-art (SOTA) architecture of general object detectors.

We consider face detector as a special task of general objector detection. General target detection is aimed at multiple categories, while face detection is a dichotomous problem that only detects the face category. In this paper, we design a face detector based on YOLOv5 [11] which has been verified for its superior performance in general target detection tasks. To resolve the challenge of multiscale, small faces, low-light, and dense scenes, we optimized the model with some practical tricks. We also use superresolution reconstruction technology [13] for processing false detection of fuzzy small-scale faces, contributing to richer texture information and improves the authenticity of visual perception. The algorithm proposed in the paper is called SR-YOLOv5, which guarantees the detection speed while improving the detection accuracy of small targets.

## 2. Related Work

In this section, we introduce the related work from three following parts. First, we review recent progress on face detection in low-resolution conditions. Second, we give an overall description of the YOLO series. Third, we describe the principle of the SR network.

### 2.1. Face Detection

Face detection has received much attention due to its wide practical applications [14]. Before deep convolutional neural network (deep CNN) was widely used, hand-made features were a very important part of face detectors. Researchers proposed many robust hand-made features [15], such as HAAR [16], HOG [17], LBP [18], SIFT [19], DPM [20], and ACF [21]. However, the performance of these feature extractors has been far surpassed by deep CNN. In recent years, numerous models have emerged, and deep CNN has shown excellent performance in general target detection tasks. The target detection task is modeled as two problems of classification and regression of target candidate regions. There are many object detection networks including RCNN family [2, 5, 15, 22], SSD [6], YOLO series [7–11], FPN [23], MMDetection [24], EfficientDet [25], transformer (DETR) [26], and Centernet [22].

From the multiscale, small face, low light, dense scene, and other challenges encountered in face detection, face detection is the same as general target detection. Thus, face detection networks can learn from general object detection networks. There are also some specific problems containing scale, pose, occlusion, expression, and makeup. Many researchers developed methods to deal with the above problems, such as Cascade CNN, MTCNN, HR, and SSH. They also test their algorithm on public datasets [27].

### 2.2. SR

In the actual application scene, some images will be fuzzy and of low quality because of the limitation of environment and shooting technology. Such images have poor performance in the region of interest (RoI). Therefore, the researchers proposed the image superresolution reconstruction technology to enrich the detailed information of low-resolution images and improve the expression ability of images. Currently, superresolution reconstruction technology [13] based on deep learning is widely used. Among them, the superresolution image generated by the Generative Adversarial Networks (GAN) [12] has a better visual effect, which is called SRGAN. By training a generation function, SRGAN converts the input low-resolution image into the corresponding superresolution image [28]. Based on SRResNet, SRGAN uses perceptual loss and adversarial loss to make the generated images closer to the target images.

The SRGAN network is composed of a generator and a discriminator, and its network model is shown as in Figure 1 [13] below. The core of the generator network is multiple residual blocks, each residual block containing two 3 × 3 convolutional layers. After the convolutional layer is a batch normalization layer, PReLU is used as the activation function [29]. The discriminant network uses a network structure similar to VGG-19, but without maximum pooling. The discriminant network contains eight convolutional layers. As the number of network layers increases, the number of features increases, and the size of features decreases. Leaky ReLU acts as an activation function. Finally, the network uses two full convolution layers and a sigmoid activation function to capture the potentiality of the learned real sample, which is used to determine whether the image comes from the high-resolution image of the real sample or the superresolution image of the fake sample.

### 2.3. YOLO

In the past five years, the YOLO algorithm has been transformed into the fifth version with many innovative ideas from the object detection community. The first three versions including YOLOv1 [7], YOLOv2 [8], and YOLOv3 [9] were all proposed by the author of the original YOLO algorithm, and YOLOv3 [9] is recognized as a milestone with big improvements in performance and speed. We can find multiscale features (FPN) [23], a better backbone network (Darknet53), and replacing the soft-max loss with the binary cross-entropy loss in this algorithm.

YOLOv4 [10] was released by a different research team in early 2020. The team explored a lot of options in almost all aspects of the YOLOv3 [9] algorithm, including the backbone, and what they call bags of freebies and bags of specials. One month later, the YOLOv5 [11] was released by another different research team which significantly reduced size, increased in speed [10], and had a full implementation in Python (PyTorch). It is welcome by the object detection community until now.

YOLOv5 using CSPDarknet as a network of feature extraction, target information is extracted from the input image. The combination of CSP and Darknet formed the CSPDarknet.  Figure 2 shows the structure of CSPDarknet. For the input tensor, CSP divides it into two parts in the channel, one part is convoluted once, the other part is convolution-residuals multiple times. The tensor is obtained by multiple convolution-residual operations, and the tensor obtained by one convolution of the previous part is spliced in channel dimensions. CSP makes the output graph retain more network gradient information and maintains the performance of the network while reducing the computational effort.

In the operation, the features of the previous stage can be used as the input of the next stage for up-sampling or down-sampling, and at the same time, the CONCAT with the feature map of the same size in the main part. This pyramid structure makes the high-level feature map integrate the accurate position information of the low level [30] and improves the accuracy of regression.

During detection, the input tensor is divided into *S* × *S* grids, and any one of the grids will be responsible for detecting the target if the center point of the target is located in it. For each grid, there will be B anchors. Specifically, for each anchor frame, (5 + *C*) values are predicted, with the first 5 values used to regress anchor's center point position, the size of the anchor frame, then to determine whether there is a target. *C* is the total number of target categories. If the center of the target is in this grid, then the target will be acquired and judge whether it is a human face. The position of the regression box of the target can be obtained by the following formula:

(1) $$\begin{array}{c} \;C_{i}^{j}=P_{i,j}*{\text{IOU}}_{\text{pred}}^{\text{truth}}. \end{array}$$

In the above parameters, *i* and *j* represent the *j*th regression box of the *i*th grid, *C*_*i*_^*j*^ represents the confidence score of the *j*th bounding box of the *i*th grid. *P*_*i*,*j*_ represents whether there is a target, if the target is in the *j*th box, the value of *P*_*i*,*j*_ = 1; otherwise, *P*_*i*,*j*_ = 0. The IOU_pred_^truth^ is a widely used parameter that represents the intersection over union between the predicted box and ground truth box [31]. The higher the IOU score, the more accurate the position of the predicted box.

### 2.4. Loss Function of YOLOv5s

The loss function can be expressed as follows:

(2) $$\begin{array}{c} \text{loss}=l_{\text{box}}+l_{\text{cls}}+l_{\text{obj}}, \end{array}$$

where  *l*_box_, *l*_cls_, and *l*_obj_ are bounding box regression loss function, classification loss function, and confidence loss function, respectively.

The bounding box regression loss function is defined as

(3) $$\begin{array}{c} l_{\text{box}}=\lambda_{\text{coord}}\;\overset{S^{2}}{\underset{i=0}{\sum }}\overset{B}{\underset{j=0}{\sum }}I_{i,j}^{\text{ojb}}bj\left(2-w_{i}\times h_{i}\right)\;\left[{\left(x_{i}-{\overset{\wedge }{x}}_{i}^{j}\right)}^{2}+{\left(y_{i}-{\overset{\wedge }{y}}_{i}^{j}\right)}^{2}+{\left(w_{i}-{\overset{\wedge }{w}}_{i}^{j}\right)}^{2}+{\left(h_{i}-{\overset{\wedge }{h}}_{i}^{j}\right)}^{2}\right]. \end{array}$$

The classification loss function is defined as

(4) $$\begin{array}{c} l_{\text{cls}}=\lambda_{\text{class}}\overset{S^{2}}{\underset{i=0}{\sum }}\overset{B}{\underset{j=0}{\sum }}I_{i,j}^{\text{obj}}\underset{C\in \text{classes}}{\sum }p_{i}\left(c\right)\log\left({\hat{p}}_{l}\left(c\right)\right). \end{array}$$

The confidence loss function is defined as

(5) $$\begin{array}{c} l_{\text{obj}}=\lambda_{\text{noobj}}\overset{S^{2}}{\underset{i=0}{\sum }}\overset{B}{\underset{j=0}{\sum }}I_{i,j}^{\text{noobj}}{\left(c_{i}-{\overset{\wedge }{c}}_{l}\right)}^{2}+\lambda_{\text{obj}}\overset{s^{2}}{\underset{i=0}{\sum }}\overset{B}{\underset{j=0}{\sum }}I_{i,j}^{\text{obj}}{\left(c_{i}-{\overset{\wedge }{c}}_{l}\right)}^{2}, \end{array}$$

where *λ*_coord_ is the position loss coefficient, *λ*_class_ is the category loss coefficient, $\hat{x}$, $\hat{y}$is the true central coordinate of the target, and $\hat{w}$, $\hat{h}$ is the width and height of the target.

If the anchor box at (*i*, *j*) contains targets, then the value *I*_*i*,*j*_^obj^ is 1; otherwise, the value is 0. *p*_*i*_(*c*) represents the category probability of the target, and ${\hat{p}}_{l}\left(c\right)$ is the true value of the category. The length of the two is equal to the total number of categories *C*.

## 3. Method

This paper focuses on improving the detection accuracy of small faces in surveillance images. Because of the comparison of the four versions of YOLOv5 including YOLOv5m, YOLOv5l, YOLOv5x, and YOLOv5s, the YOLOv5s model is smaller and easier to deploy quickly. Therefore, our research is based on the YOLOv5s model. We optimize the backbone, then integrate image superresolution technology on the head and improve the loss function to ensure efficient detection speed.

### 3.1. SR-YOLOv5

#### 3.1.1. Adaptive Anchor

The calculation of adaptive anchor is added in YOLOv5s. Before each training, the *K*-means algorithm is used to cluster the ground truth of all samples in the training set and to find out the optimal group of anchor point frames in the high complexity and high recall rate. The results of anchor boxes clustered by the algorithm are shown in Table 1.

#### 3.1.2. Network Architecture

*(1) Backbone*. The overall architecture of improved YOLOv5s is depicted in Figure 3 which consists of the backbone, detection neck, and detection head. Firstly, a newly designed backbone named CSPNet is used. We change it with a new block called CBS consists of Conv layer, BN layer, and a SILU [32]. Secondly, a stem block is used to replace the focus layer in YOLOv5s. Thirdly, a C3 block is used to replace the original CSP block with two halves. One is passed through a CBS block, some bottleneck blocks, and a Conv layer, while another consists of a Conv layer. After the two paths with a CONCAT and a CBS block followed, we also change the SPP block [4] to improve the face detection performance. In this block, the size of the three kernels is modified to smaller kernels.

*(2) Detection Neck*. The structure of the detection neck is also shown in Figure 3 which consists of a normal feature pyramid network (FPN) [23] and path aggregation network (PAN) [3]. However, we modify the details of some modules, such as the CS block and the CBS block we proposed.

*(3) Detection Head*. Through feature pyramid structure and path aggregation [33] network, the front segment of the network realizes the full fusion of low-level features and high-level features to obtain rich feature maps, which can detect the most high-resolution face samples. However, for low-resolution images, feature fusion cannot enhance the original information of the image, and through layers of iteration, the prior information of small faces is still lacking. To enhance the detection rate of small faces in low-resolution images, SR is fused in the detection head part of the network. For the grid to be determined, the region information is input into SRGAN to carry out superresolution reconstruction and face detection again through its coordinate information. Finally, the output of the two-stage face detector is integrated and output.

### 3.2. Loss Function

IOU is a frequently used index in target detection. In most anchor-based [34] methods, it is used not only to judge the positive and negative sample but also to assess the distance between the location of the predicted box and the ground truth. The paper proposes that a regression positioning loss [35] should be considered: overlapping area, center point distance, and aspect ratio, which have aroused wide concern. At present, more and more researchers propose better performance algorithms, such as IOU, GIOU, DIOU, and CIOU. In this paper, we propose to replace GIOU in YOLOv5s with CIOU and nonmaximal suppression (NMS).

Our bounding box regression loss function is defined as

(6) $$\begin{array}{c} l_{\text{box}}^{\prime }=1-\text{IOU}+\frac{\rho^{2}\left(b,\hat{b}\right)}{c^{2}}+\frac{16}{\pi^{4}}\frac{{\left(\arctan\left(\overset{\wedge }{w}/\overset{\wedge }{h}\right)-\arctan\left(w/h\right)\right)}^{4}}{1-\text{IOU}+\left(4/\pi^{2}\right){\left(\arctan\left(\overset{\wedge }{w}/\overset{\wedge }{h}\right)-\arctan\left(w/h\right)\right)}^{2}}, \end{array}$$

where *b*, *b*′ represents the center point of the box, *ρ* represents the Euclidean distance, *c* represents the diagonal distance of the minimum enclosing rectangle, and $\hat{\text{w}}$, $\hat{h}$ is the width and height of the target.

In surveillance video images [36], face targets are not only numerous but also stacked, which leads to more than one target in each grid. However, judging by a single threshold often leads to a low recall rate [37]. Therefore, through the combination of CIOU and NMS, the candidate box in the same grid can be judged and screened several times through the cyclic structure, which can effectively avoid the problem of missed detection.

## 4. Experiments

### 4.1. Dataset and Experimental Environment Configuration

This experiment uses a face detection benchmark called wider face [27], which is recognized as the largest one among public available datasets. The details of publicly available datasets are shown in Table 2. These faces in the wider face dataset have great changes in scale, posture, and occlusion with an average of 12.2 faces per image, and there are many dense small faces. The dataset contains three parts: training set, validation set, and test set, accounting for 40%, 10%, and 50% of the sample number, respectively. This paper focuses on the detection of small faces, which will be more difficult to detect. Therefore, the verification set and test set are divided into three difficulty levels: easy, medium, and hard. There are many small-scale faces in the hard subset, most of which are 10 pixels~50 pixels. Thus, this benchmark is suitable to verify the effectiveness and performance in realistic scenes. The experimental environment configuration is shown in Table 3.

### 4.2. Training and Testing of SR-YOLOv5 Models

#### 4.2.1. Training Model

The YOLOv5s code [11] is used as our basic framework, and we implement all the modifications as described above in PyTorch. We set the initial learning rate at 1*E*-2, and then we go down to 1*E*-5 with the decay rate of 5*E*-3. We set momentum at 0.8 in the first 20 epochs. After that, the momentum is 0.937. The precision-recall (PR) curves of our SR-YOLOv5 detector are shown in Figure 4.

#### 4.2.2. Testing Model

The detection effect of our improved algorithm on the wider face dataset is shown in Figure 5. It can be seen that this method has good robustness and high accuracy for small faces in various complex scenes. (a) The figure can detect faces with slight occlusion. (b) The figure itself has a low resolution, but the detection result shows that the detection effect is still good. (c) The figure fully shows that numerous small faces can be well detected even in a high-density crowd.

### 4.3. Evaluation Index

In the evaluation of the effect of face detection, there are some relevant parameters: TP (true positives) means that the face is detected, and there are faces in the actual picture; TN (true negatives) means that no face is detected, and no face exists in the actual picture; FP (false positives) means that faces are detected when there is no face in the actual image. FN (false negatives) means that no face is detected, but there are faces in the actual image. The evaluation indexes of the model in this paper include recall rate *R*, accuracy rate *P*, and *F*_1_ score. The recall rate is used to evaluate the proportion of faces detected to the total face price in the sample. The accuracy rate is used to evaluate the proportion of the correct face detected in the total face detected, When the two are close, refer to *F*_1_ score, and the higher the score of *F*_1_, the better the algorithm will be.

(7) $$\begin{array}{c} P=\frac{\text{TP}}{\text{TP}+\text{FP}}, \end{array}$$

(8) $$\begin{array}{c} R=\frac{\text{TP}}{\text{TP}+\text{FN}}, \end{array}$$

(9) $$\begin{array}{c} F_{1}=\frac{2\times P\times R}{P+R}. \end{array}$$

The trained model is verified on the validation set, and the recall rate *R* = 0.96, accuracy rate *P* = 0.975, and *F*_1_ = 96.75 were obtained from Equations (6), (8), and (9). From the point of view of the score, the proposed algorithm has better performance.

### 4.4. Model Performance Analysis

After the fusion of SRGAN in the YOLOv5 network, the rationality and effectiveness of the fused network should be verified first. We select 1000 pictures from the test set for network model test and comparison. As shown in Table 4, compared with YOLOv3, the speed of the network after the fusion of superpartition reconstruction technology is reduced, because the network depth is increased when the new network is integrated. Compared with the HR using Resnet101 as the backbone network, the average detection accuracy of the improved network has been significantly improved, which is 2.3% higher than HR.

### 4.5. Comparison of Accuracy of Relevant Algorithms

To demonstrate the effectiveness of the algorithm, some excellent face detection algorithms are selected to test on the wider face dataset, and the results are analyzed. As shown in Table 5, all existing methods achieve mAP in a range of 85.1-95.6% on the easy subset, 82.0-94.3% on the medium subset, and 62.9-85.3% on the hard subset. The mean average precision of the proposed algorithm on the easy, medium, and hard validation subsets are 96.3%, 94.9%, and 88.2%, respectively, which is 0.7%, 0.6%, and 2.9% higher than the top one.

The SR-YOLOv5 proposed in this paper is improved on the YOLOv5s network, and the image superresolution reconstruction technology is introduced for the secondary detection of small-scale fuzzy faces, deepening the network to make facial features easier to be detected, capturing small target information, and making the network more accurate when processing complex face and nonface classification and detection. Through the comparative experiment on the wider face dataset, it is verified that the method used in this paper has higher detection accuracy and better robustness, especially in the hard subset, it has more outstanding performance.

## 5. Conclusion

To improve the face detection rate of security surveillance scenes with diverse scales in dense face images, this paper proposes a small face detection algorithm suitable for complex scenes. We integrate the image superresolution reconstruction technology into the network structure of the target detection algorithm YOLOv5s. YOLOv5s has a fast detection speed, but its detection accuracy is reduced compared with other SOTA detection algorithms. SRGAN is used to improve the performance of the detection head and then improve the detection accuracy of small-scale fuzzy faces in complex scenes. In the same environment with other face detection algorithms, using the same dataset to carry out comparative experiments, the results confirm the feasibility and superiority of the proposed method.

## Figures and Tables

**Figure 1:** SRGAN network model.

**Figure 2:** Structures of YOLOv5s.

**Figure 3:** The architecture of improved SR-YOLOv5.

**Figure 4:** Precision-recall (PR) curves of our SR-YOLOv5 detector.

**Figure 5:** Part of the test results.

**Table 1:** Results of anchor boxes of the training set.

Feature map	Size	Anchor
Predict one	13 × 13	(43, 59) (76, 89) (178, 234)
Predict two	26 × 26	(30, 36) (22, 26) (15, 18)
Predict three	52 × 52	(10, 12) (7, 9) (5, 6)

**Table 2:** Available datasets.

Datasets	Pictures	Faces
Wider face	32203	393703
AFW	205	473
FDDB	2845	5171
Pascal face	851	1341
IJB-A	24327	49759
MALF	5250	11931

**Table 3:** Experimental environment configuration.

Experimental environment	Configuration
Operating system	Linux 64
GPU	TITAN Xp
CPU	Intel(R)Core i7-3770CPU@
Deep learning framework	PyTorch

**Table 4:** Performance comparison using different models.

Model	Backbone	AP50	Time/ms
HR	Resnet101	57.5%	198
YOLOv3	Darknet53	57.9%	51
Ours	YOLOv5s-SRGAN	59.8%	75

**Table 5:** Comparison of mAP using different face detection algorithms.

Face detection algorithms	Easy	Medium	Hard
MTCNN	85.1%	82.0%	62.9%
CMS-RCNN	90.2%	87.4%	64.3%
HR	92.5%	91.0%	81.9%
S3FD	93.7%	92.5%	85.9%
TinaFace	95.6%	94.3%	85.3%
Ours	96.3%	94.9%	88.2%

## Data Availability

The data (wider face dataset) used in this research is cited in the references.

## References

[1] Zou Z., Shi Z., Guo Y., Ye J. (2019). Object detection in 20 years: a survey. https://arxiv.org/abs/1905.05055.

[2] Ren S., He K., Girshick R., Sun J. (2015). Faster r-cnn: towards real-time object detection with region proposal networks. *Advances in Neural Information Processing Systems*.

[3] Liu S., Qi L., Qin H., Shi J., Jia J. Path aggregation network for instance segmentation.

[4] He K., Zhang X., Ren S., Sun J. (2015). Spatial pyramid pooling in deep convolutional networks for visual recognition. *IEEE Transactions on Pattern Analysis and Machine Intelligence*.

[5] He K., Gkioxari G., Dollár P., Girshick R. Mask r-cnn..

[6] Liu W., Anguelov D., Erhan D. (2016). Ssd: single shot multibox detector. *Computer Vision – ECCV 2016*.

[7] Redmon J., Divvala S., Girshick R., Farhadi A. You only look once: unified, real-time object detection.

[8] Redmon J., Farhadi A. YOLO9000: better, faster, stronger.

[9] Redmon J., Farhadi A. (2018). Yolov3: an incremental improvement. https://arxiv.org/abs/1804.02767.

[10] Bochkovskiy A., Wang C. Y., Liao H. Y. M. (2020). Yolov4: optimal speed and accuracy of object detection. https://arxiv.org/abs/2004.10934.

[11] Ultralytics (2021). Yolov5. https://github.com/ultralytics/yolov5.

[12] Deng J., Guo J., Zhou Y., Yu J., Kotsia I., Zafeiriou S. (2019). Retinaface: single-stage dense face localization in the wild. https://arxiv.org/abs/1905.00641.

[13] Ledig C., Theis L., Huszár F. Photo-realistic single image super-resolution using a generative adversarial network.

[14] Xu C., Gao Z., Zhang H., Li S., de Albuquerque V. H. C. (2021). Video salient object detection using dual-stream spatiotemporal attention. *Applied Soft Computing*.

[15] Qi D., Tan W., Yao Q., Liu J. (2021). YOLO5Face: why reinventing a face detector. https://arxiv.org/abs/2105.12931.

[16] Lienhart R., Maydt J. An extended set of haar-like features for rapid object detection.

[17] Dalal N., Triggs B. Histograms of oriented gradients for human detection.

[18] Ahonen T., Hadid A., Pietikainen M. (2006). Face description with local binary patterns: application to face recognition. *IEEE Transactions on Pattern Analysis and Machine Intelligence*.

[19] Long J., Shelhamer E., Darrell T. Fully convolutional networks for semantic segmentation.

[20] Zheng L., Shen L., Tian L., Wang S., Wang J., Tian Q. Scalable person re-identification: a benchmark.

[21] Hwang S., Park J., Kim N., Choi Y., So Kweon I. Multispectral pedestrian detection: benchmark dataset and baseline.

[22] Cai Z., Vasconcelos N. Cascade r-cnn: delving into high-quality object detection.

[23] Lin T. Y., Dollár P., Girshick R., He K., Hariharan B., Belongie S. Feature pyramid networks for object detection.

[24] Chen K., Wang J., Pang J. (2019). MMDetection: open mmlab detection toolbox and benchmark.. https://arxiv.org/abs/1906.07155.

[25] Tan M., Pang R., Le Q. V. Efficientdet: scalable and efficient object detection.

[26] Carion N., Massa F., Synnaeve G., Usunier N., Kirillov A., Zagoruyko S. (2020). End-to-end object detection with transformers. *Computer Vision – ECCV 202*.

[27] Yang S., Luo P., Loy C. C., Tang X. Wider face: a face detection benchmark.

[28] Wang C., Dong S., Zhao X., Papanastasiou G., Zhang H., Yang G. (2016). SaliencyGAN: deep learning semi-supervised salient object detection in the fog of IoTC. *IEEE Transactions on Industrial Informatics*.

[29] Jiang T., Cheng J. Target recognition based on CNN with LeakyReLU and PReLU activation functions.

[30] Liu S., Han K., Song Z., Li M. Texture characteristic extraction of medical images based on pyramid structure wavelet transform.

[31] Huang C., Zong Y., Chen J., Liu W., Lloret J., Mukherjee M. (2021). A deep segmentation network of stent Structs based on IoT for interventional cardiovascular diagnosis. *IEEE Wireless Communications*.

[32] Elfwing S., Uchibe E., Doya K. (2018). Sigmoid-weighted linear units for neural network function approximation in reinforcement learning. *Neural Networks*.

[33] Bai H., Cheng J., Huang X., Liu S., Deng C. (2021). HCANet: a hierarchical context aggregation network for semantic segmentation of high-resolution remote sensing images. *IEEE Geoscience and Remote Sensing Letters.*.

[34] Yu B., Tao D. (2019). Anchor cascade for efficient face detection. *IEEE Transactions on Image Processing*.

[35] Chen C., Yang X., Huang R. Region proposal network with graph prior and IoU-balance loss for landmark detection in 3D ultrasound.

[36] Ding C., Tao D. (2018). Trunk-branch ensemble convolutional neural networks for video-based face recognition. *IEEE Transactions on Pattern Analysis and Machine Intelligence*.

[37] Tang Z., Zhao G., Ouyang T. (2021). Two-phase deep learning model for short-term wind direction forecasting. *Renewable Energy*.

